# The Association of Sperm DNA Fragment and Assisted Reproductive Outcomes: A Meta-Analysis

**DOI:** 10.1155/2022/1126616

**Published:** 2022-09-14

**Authors:** Yue Chen, Wei Li, Xin Chen

**Affiliations:** ^1^Department of Laboratory Medical Center, PLA North Military Command Region General Hospital, Shenyang 110000, China; ^2^Department of Emergency, Central South University Xiangya School of Medicine Affiliated Haikou Hospital, Haikou 570208, China; ^3^Department of Laboratory, General Hospital of the Northern Theater of the Chinese People's Liberation Army, Shenyang 110000, China

## Abstract

**Objective:**

To analyze the effect of sperm DNA fragmentation index (DFI) on the outcomes of in vitro fertilization (IVF) and intracytoplasmic sperm injection (ICSI).

**Methods:**

Literature search was conducted on English databases PubMed, Cochrane, and Embase to obtain eligible studies.

**Results:**

A total of 11 cohort studies were included and analyzed using the random effects model. The results illustrated that the IVF fertilization rate (RR = 0.94, 95% CI: 0.77-1.14, *P* = 0.61), pregnancy rate (RR = 0.83, 95% CI: 0.57-1.21, *P* = 0.32), and live birth rate (RR = 0.53, 95% CI: 0.16-1.80, *P* = 0.31) in the high DFI group were statistically insignificant with those in the low FI group. The correlations between DFI and ICSI fertilization rate (RR = 0.79, 95% CI: 0.52-1.18, *P* = 0.25), pregnancy rate (RR = 0.89, 95% CI: 0.74-1.06, *P* = 0.18), and live birth rate (RR = 0.89, 95% CI: 0.70-1.14, *P* = 0.36) were also not statistically significant.

**Conclusion:**

This study has observed no significant correlation between sperm DFI and assisted reproductive outcomes. Multicenter large-sample clinical trials are required to conclusively determine the impact of DNA damage on the clinical outcomes of assisted reproduction.

## 1. Introduction

Infertility is a worldwide health problem that has an incidence of about 7%-15% [1]. In recent years, with the continuous development of medical technology, assisted reproductive technology (ART), including intrauterine artificial insemination (IUI), in vitro fertilization (IVF), and intracytoplasmic sperm injection (ICSI), has brought new options to infertile couples. Among the causes of infertility symptoms, male factors such as oligospermia, low sperm motility, and abnormal sperm morphology lead to approximately the same rate of infertility as female factors such as endometriosis and blocked fallopian tubes [2]. In particular, merging data have shown that male sperm disorders were drastically associated with clinical outcomes in ART [2].

As the carrier of human genetic material, sperm DNA plays a crucial role in human reproduction and survival by transferring genetic material to offspring completely. Since sperm has no repair mechanisms, DNA damage is present in almost all sperms. Whether sperm DNA damage has an adverse impact on reproductive outcomes is a question of particular clinical concern [3]. Studies have shown that the integrity of sperm DNA has a significant correlation with the decline of female natural pregnancy rate and male infertility [4]. At present, the pregnancy rate of IVF and intracytoplasmic sperm injection is low. Therefore, it is increasingly necessary to develop techniques to accurately diagnose sperm damage and predict the impact on the clinical results of assisted reproduction [5]. With the continuous development and improvement of sperm detection technology, emerging methods to detect the integrity of sperm chromatin have been established, including comet assay, sperm chromatin diffusion assay (SCD), terminal transferase-mediated dUTP terminal labelling (TUNEL), sperm chromatin structure analysis (SCSA), and acridine orange test. Currently, the SCSA is considered the “gold standard” for sperm DNA integrity detection.

Therefore, this study is aimed at exploring the impact of sperm DNA fragment index on assisted reproduction through literature retrieval and meta-analysis. The detection method of sperm integrity is limited to “gold standard” chromatin structure analysis.

## 2. Methods

### 2.1. Bibliography Retrieval

The English databases PubMed, Cochrane, and Embase were searched from January 2000 to March 2022. The search method was medical subject headings combined with free words. The search items included “in-vitro fertilization OR IVF OR intracytoplasmic sperm injection OR ICSI OR assisted reproductive technique OR ART” AND “Sperm DNA damage OR sperm DNA fragmentation OR DNA fragmentation index OR DFI” AND “sperm chromatin structure assay OR SCSA.”

### 2.2. Literature Screening

The following are the inclusion criteria: (1) subjects with normal ovarian reserve function receiving IVF or ICSI; (2) stratification of patients into the low- and high-DFI groups; (3) outcome measures including at least one of the following: IVF/ICSI fertilization rate, pregnancy rate, or live birth rate; (4) prospective or retrospective cohort study; and (5) DFI detection by SCSA.

The following are the exclusion criteria: (1) DFI not detected by SCSA; (2) ART other than IVF or ICSI; (3) news reports, expert opinions, critical literature, and abstracts; (4) republished literature; (5) incomplete data information or insufficient literature available for data analysis; (6) DIF threshold not clearly defined; and (7) unavailable full text.

### 2.3. Document Data Extraction

Two researchers conducted literature search and screened potentially eligible studies according to the inclusion/exclusion criteria. The following relevant data were extracted, including title, publication date, author's name, research type, study population, intervention measures, outcome measures, research methods, and subject characteristics. Any disagreements were resolved by discussion and arbitration by another independent senior author.

### 2.4. Literature Quality Evaluation

The NHLBI-NIH guidelines (http://www.nhlbi.nih.gov/health-topics/study-quality-assessment-tools) were applied to evaluate the quality of the included studies. The quality assessment tool contained 14 questions with an answer of “yes/no” for each item. On a scale of 14 points, higher score indicated better quality. Two researchers independently evaluated the quality of the included literature before cross-checking. Discrepancies were settled by consulting a third researcher.

### 2.5. Statistical Method

The Cochrane software RevMan5.4 was utilized for data analysis. The categorical data were compared using the relative risk (RR) coefficient with 95% confidence interval. Interstudy heterogeneity was evaluated using the chi-square test and the *I*^2^ statistic, with *I*^2^ > 50% denoting significant heterogeneity. The RR was calculated with the fixed or random effects model depending on the heterogeneity assessment. Egger's test and funnel plot were consulted to estimate possible publication bias. A two-sided *P* value < 0.05 denoted statistical significance.

## 3. Results

### 3.1. Literature Search Results

2132 relevant literatures were obtained through database retrieval in this study. After exclusion of duplicate publications, the study title and abstracts were screened for eligibility. Finally, a total of 12 publications were finally included in this meta-analysis. The specific screening process and results are shown in Figure 1.

### 3.2. Characteristics and Quality Evaluation

The basic information of the 12 included English literatures [6–17] is shown in Table 1. All these were cohort studies published between 2005 and 2020, of which 4 were retrospective, 5 were prospective, and 3 were bidirectional cohort studies. Five articles reported using both ICSI and IVT, whereas 5 and 1 publication employed only ICSI and IVT, respectively. The other 6 papers studied both ICSI and IVT techniques. The DFI threshold defined varied across studies, with an overall range of 15% -30%. A total of 5, 7, and 3 studies reported IVT fertilization rate, pregnancy rate, and live birth rate, respectively. There were 5, 10, and 3 articles reported ICSI fertilization rate, pregnancy rate, and live birth rate, respectively. The total score of NHLBI-NIH were 8-10 points, with only 1 scored 5 points. The scoring results are shown in Table 1. The quality of the included literature was evaluated to be high.

### 3.3. Meta-analysis Results

#### 3.3.1. Correlation between DFI and IVF Clinical Outcomes

Patients were divided into the high- and low-DFI groups, using the boundary value as the DFI threshold. The heterogeneity assessment of the IVF fertilization rate, pregnancy rate, and live birth rate was *I*^2^ = 55%, 73%, and 76%, respectively. Significant heterogeneity was noted, for which the random effects model was applied. The results of the meta-analysis showed that the IVF fertilization rate in the high DFI group was statistically insignificant with that in the low DFI group (RR = 0.94, 95% CI: 0.77-1.14, *Z* = 0.51, *P* = 0.61), as shown in Figure 2. Similarly, the IVF pregnancy rate in both groups was also insignificant (RR = 0.74, 95% CI: 0.50-1.12; *Z* = 1.47, *P* = 0.14) (Figure 3). The IVF live yield in the high DFI group was also insignificant with that in the low DFI group (RR = 0.53, 95% CI: 0.16-1.80; *Z* = 1.01, *P* = 0.31) (Figure 4). However, the IVF pregnancy rate and live birth rate in the high DFI group were significantly lower than those in the DFI when the fixed effects model was used.

#### 3.3.2. Correlation between DFI and ICSI Clinical Results

No significant differences with regard to ICSI fertilization rate, pregnancy rate, and live birth rate were noted between the high- and low- DFI groups. The correlation between DFI and ICSI fertilization rate, pregnancy rate, and live birth rate were RR = 0.79 (95% CI: 0.52-1.18, *P* = 0.25, Figure 5), RR = 0.90 (95% CI: 0.76-1.07, *P* = 0.24, Figure 6), and RR = 0.89 (95% CI: 0.70-1.14, *P* = 0.36, Figure 7), respectively.

#### 3.3.3. Publication Bias Analysis

Funnel plots were drawn for the study groups with ≥5 included literatures. The results showed that the included literatures were distributed symmetrically around the combined effect RR value, suggesting no significant publication bias (*P* > 0.05), as shown in Figures 8–11. Similarly, Egger's test performed for groups with <5 included articles also showed no publication bias (*P* > 0.05).

## 4. Discussion

Currently, studies that analyzed the relationship between sperm DNA damage and clinical outcomes following IVF and intracytoplasmic sperm injection reported inconsistent findings. There is still ongoing controversy regarding the impact of DNA loss on ART results. Some studies [18, 19] have suggested that sperm DNA integrity affects the success rate of clinical pregnancy by influencing fertilization and embryonic development. A retrospective cohort study conducted by Boe-Hansen et al. [6] in 2006 showed that the clinical pregnancy rate in IVF decreased in the presence of severe DNA damage. In comparison, other studies [20, 21] reported no correlation between DFI and IVF outcomes. For instance, studies by Niu et al. [13] have demonstrated that the DFI index had no significant influences on IVF fertilization rate, clinical pregnancy rate, or delivery rate, and high DNA fragmentation was only related to low embryo quality. Although a high degree of DNA fragmentation does not necessarily affect fertilization rates, once the embryonic genome is activated, the consequences of damaged paternal DNA can manifest possibly triggering apoptosis, leading to early postimplantation miscarriage [22]. DFI values in some spontaneous abortion groups seem to support this hypothesis, but there is some debate about the effect of DFI on ICIS. Some scientists believe that sperm DNA integrity will affect the clinical outcome of ICIS. Miciński et al. [12] indicated that sperm DNA fragmentation might be related to the pregnancy rate after ICSI. Speyer et al. [14] observed that when DNA fragmentation increased, the fertilization rate in the ICSI cycle would decrease correspondingly. Moreover, unfavorable clinical outcomes in terms of fertilization rate, pregnancy rate, and live birth rate in patients with high levels of sperm DNA fragmentation were also reported [7]. Others, however, have suggested that DNA integrity had no impact on the clinical outcome of ICIS. For example, the retrospective cohort study conducted by Yang et al. [15] in 2019 illustrated no significant differences in fertilization, embryo quality, pregnancy rate, or abortion in ICSI related to DNA damage. The prospective cohort study conducted by Green et al. [11] in 2020 also reached a similar conclusion. Despite numerous studies discussing the relationship between DFI and pregnancy rates [23–25], sperm chromatin testing as part of the assessment of male fertility potential is still not widely accepted. The reasons for this are many, chiefly the lack of standardized protocols for reproducible results and the fact that thresholds in many trials have not been validated. Furthermore, the limitations of our understanding of the underlying nature of DFI and the lack of sufficient data demonstrate the relationship between DFI and reproductive outcomes after IVF and/or ICSI.

The 12 literatures were included in this meta-analysis. The overall quality is high, and the selectivity bias is limited. At present, SCSA is considered to be the “gold standard” for sperm DNA integrity detection, which was adopted as the criteria for inclusion. The heterogeneity test results of the included studies showed heterogeneity in parameters except for the ICSI pregnancy rate, for which the fixed effects model was used for analysis. The meta-analysis results illustrated that the IVF fertilization rate, pregnancy rate, and live birth rate of high DIF were statistically insignificant with those in the IVF group. Differences regarding IVF fertilization rate, pregnancy rate, and live birth rate in the ICSI group were also insignificant. Therefore, this study showed that sperm DNA fragments did not significantly correlate with IVF/ICSI fertilization rate, pregnancy rate, and live birth rate.

This study suffered from several limitations. First, because the included literature included men and women with assisted reproductive age between 30 and 35 years of age, age-considered subgroup analyses were not considered. Secondly, the fact that only studies using SCSA for DFI detection was included may introduce biases that might not reflect the impact of the overall DNA fragment index on assisted reproductive outcomes. This study concluded that no differences were observed in sperm DFI in assisted reproductive outcomes. Although the threshold between high DFI and low DFI is concentrated at 15%-30%, this range is relatively large, and multiple groups of DFI can be analyzed. In addition, SCD and TUNEL are other methods to detect sperm chromatin integrity.

In conclusion, consistent with the newly released guidelines related to DNA fragment detection [26], this study observed no significant correlation between sperm DFI and assisted reproductive outcomes. Multicenter and large sample clinical trials should to be carried out to conclusively determine the impact of DNA damage on assisted reproductive outcomes.

## Figures and Tables

**Figure 1:** Document screening process and results.

**Figure 2:** Correlation between DFI and IVF fertilization rate.

**Figure 3:** Correlation between DFI and IVF pregnancy rate.

**Figure 4:** Correlation between DFI and IVF live birth rate.

**Figure 5:** Correlation between DFI and ICSI fertilization rate.

**Figure 6:** Correlation between DFI and ICSI pregnancy rate.

**Figure 7:** Correlation between DFI and ICSI live birth rate.

**Figure 8:** Funnel diagram of the correlation between DFI and IVF fertilization rate.

**Figure 9:** Funnel diagram of the correlation between DFI and IVF pregnancy rate.

**Figure 10:** Funnel diagram of the correlation between DFI and ICSI fertilization rate.

**Figure 11:** Funnel diagram of a correlation between DFI and ICSI pregnancy rate.

**Table 1:** Basic characteristics of included literature.

Author/year	Research type	ART	DFI detection method	DFI threshold	Outcome indicators	Quality score
Bungum [9]	Cohort study	ICSI and IVF	SCSA	27%	①②③④⑤⑥	8
Zini [16]	Cohort study	ICSI	SCSA	15% and 30%	⑤	8
Boe-Hansen [6]	Retrospective cohort study	ICSI and IVF	SCSA	27%	④⑤	6
Bungum [8]	Prospective cohort study	ICSI and IVF	SCSA	30%	①②③④⑤⑥	8
Miciński [12]	Prospective cohort study	ICSI	SCSA	15%	⑤	5
Speyer [14]	Cohort study	ICSI and IVF	SCSA	30%IVF 19% ICSI	①②④⑤	8
Niu [13]	Prospective cohort study	IVF	SCSA	27%	①②③	8
Bradley [7]	Retrospective cohort study	ICSI	SCSA	29%	④⑤⑥	9
Gat [10]	Retrospective cohort study	ICSI	SCSA	<15% and>30%	⑤	8
Yang [15]	Retrospective cohort study	ICSI and IVF	SCSA	15% and 30%	②⑤	8
Green [11]	Prospective cohort study	ICSI	SCSA	15%	①②	10
Jiang [17]	Prospective cohort study	ICSI and IVF	SCSA	30%	①⑤	8

① IVF fertilization rate, ② IVF pregnancy rate, ③ IVF live birth rate, ④ ICSI fertilization rate, ⑤ ICSI pregnancy rate, and ⑥ ICSI live birth rate.

## Data Availability

The data used to support the findings of this study are included within the article.
